# *PAR-2* promotes cell proliferation, migration, and invasion through activating PI3K/AKT signaling pathway in oral squamous cell carcinoma

This article has been retracted.

**DOI:** 10.1042/BSR20182476

**Published:** 2019-07-05

**Authors:** Kai-Liang Tang, Han-Ying Tang, Yi Du, Tian Tian, Shi-Jiang Xiong

**Affiliations:** 1 Department of VIP Center and Shandong Provincial Key Laboratory of Oral Biomedicine, School and Hospital of Stomatology, Shandong University, Jinan 250012, Shandong, China; 2 Department of Endodontics, Jinan Stomatological Hospital, Jinan 250001, Shandong, China; 3 Department of Oral Prosthology, Jinan Stomatological Hospital, Jinan 250001, Shandong, China; 4 Affiliated Hospital of Binzhou Medical College, Binzhou, Shandong, China

**Keywords:** Cell proliferation, Invasion, Migration, PAR-2, Oral squamous cell carcinoma, PI3K/AKT pathway

## Abstract

**Objective:** This research aimed to explore the function of protease activated receptor 2 (*PAR-2*) in oral squamous cell carcinoma (OSCC) development and progression, as well as underlying molecular mechanism.

**Methods:** Tissue samples were collected from 115 OSCC patients. Quantitative real-time PCR (qRT-PCR) was performed to measure the expression of *PAR-2* mRNA in OSCC tissues and cells. MTT and Transwell assays were used to detect the proliferation, migration, and invasion of OSCC cells, respectively. Western blot was performed to determine protein expression.

**Results:** The expression of *PAR-2* mRNA was up-regulated in OSCC tissue and cells (*P*<0.01), and its mRNA level was obviously correlated to tumor differentiation and TNM stage in OSCC (*P*<0.05 for both). The activation of *PAR-2* with PAR-2AP (*PAR-2* agonist) significantly promoted the proliferation, migration, and invasion of OSCC cells, while its knockout could inhibit malignant behaviors of OSCC cells (*P*<0.05). Excessive activation of *PAR-2* enhanced phosphorylation level of PI3K, AKT, and mTOR revealing the activation of PI3K/AKT pathway. Moreover, LY294002, the inhibitor of PI3K/AKT pathway, could reverse oncogenic action caused by *PAR-2* activation.

**Conclusion:** *PAR-2* can promote OSCC growth and progression via activating PI3K/AKT signaling pathway.

## Introduction

Oral cancer is a frequently diagnosed head and neck cancer arising from lip or oral cavity [1]. Oral squamous cell carcinoma (OSCC) accounts for more than 90% of oral cancer cases, and poses great threat to human health worldwide [2,3]. In clinic, there are some available treatments for OSCC, including surgery, radiotherapy and chemotherapy, but the prognosis of the patients is still unsatisfactory [4]. The five-year survival of OSCC patients is only approximate 50%, and the survival rate is even worse for those diagnosed at advanced stage (III or IV stage) [5,6]. Due to the lack of suitable biomarkers, most of OSCC cases have entered into advanced stages when they are first diagnosed, facing uncontrolled disease progression [7]. Therefore, to improve the management of OSCC, it is necessary to explore molecular mechanism underlying the malignancy transformation.

Protease activated receptor 2 (*PAR-2*), also known as coagulation factor II (thrombin) receptor-like 1 (F2RL1), is a transmembrane G-protein coupled receptor, belonging to the PAR family [8]. *PAR-2* can be activated by trypsin, coagulation factors tryptase and matriptase [9,10]. Abnormal activation of *PAR-2* may result in a series of pathophysiologic processes, such as inflammation, metabolism, pain processing, cardiovascular diseases, neurological disorders, and cancers [11,12]. In tumorigenesis, *PAR-2* activation may enhance biological behaviors of tumor cells, including cell proliferation, growth, invasion, and metastasis [13–15]. Oncogenic function of *PAR-2* has been reported in ovarian clear cell carcinoma [13], esophageal cancer [15], pancreatic cancer [16], hepatocellular carcinoma [17], etc. Sun et al. found that *PAR-2* might promote the migration and invasion of renal cell cancer cells through activating the PI3K/AKT signaling pathway [18]. And Al-Eryani reported that *PAR-2* could regulate the proliferation and invasion of OSCC cells *in vitro* [19]. However, molecular mechanisms underlying *PAR-2* affecting OSCC progression are rarely reported.

In the present study, we investigated expression pattern of *PAR-2* in OSCC tissues and cell lines, as well as its association with clinical characteristics of the patients. Additionally, cell experiments were constructed to explore molecular mechanisms of *PAR-2* in OSCC development and progression.

## Materials and methods

### Reagents

PAR-2 special agonist PAR-2AP, control peptide with a scrambled sequence (KGLVS-NH2), PI3K specific inhibitor LY294002 and AKT specific inhibitor MK2206 were purchased from Sigma (St Louis, MO, U.S.A.).

### Tissue samples

In the present study, 116 OSCC patients were selected from School and Hospital of Stomatology, Shandong University. None of the patients had received chemotherapy or radiotherapy before surgery. OSCC tissues and corresponding adjacent normal tissues were obtained from OSCC patients, and immediately put in liquid nitrogen. Then the tissue specimens were maintained at −80°C. In addition, clinical characteristics of the patients were collected from their medical records. The present study was approved by the Ethics Committee of the hospital. All patients signed written informed consents, and all experiments were conducted in accordance with the World Medical Association Declaration of Helsinki. The present study was approved by the ethics committee of School and Hospital of Stomatology, Shandong University (ethics approval number: ADUST160528).

### Cell culture

OSCC cells SCC-25 (ATCC® CRL-1628™) and human oral keratinocytes (HOK) (ATCC® PCS-200-014™) were purchased from American type culture collection (ATCC). All cells were cultured in 5 ml plastic flasks at a cell concentration of 4 × 10^4^ in 5 ml RPMI-1640 medium (GE Healthcare Life Sciences, Little Chalfont, U.K.) containing 10% fetal bovine serum (FBS). The cells were cultured in a humidified atmosphere at 37°C containing 5% CO_2_. Culture medium was changed every 2 days.

### RNA extraction and quantitative real-time PCR

Total RNA was extracted from tissue and cell specimens using Trizol method (TaKaRa, Japan). RNA was reversely-transcribed into cDNA via QuantiTect Reverse Transcription Kit (Qiagen, Germany) according to the instruction. Relative expression of *PAR-2* mRNA was estimated using quantitative real-time PCR (qRT-PCR) method. The reaction was performed using SYBR Premix Ex Taq™ II kit (Takara, Chiga, Japan) in 7300 Real-Time PCR System (Applied Biosystems, Foster City, CA, U.S.A.). *GAPDH* was employed as an internal normalization reference. PCR primers were as following: *GAPDH*: 5′TGCACCACCAACTGCTTAGC3′ (Forward), 5′GGCATGGACTGTGGTCATGAG3′ (reverse); *PAR-2*: 5′AGAAGCCTTATTGGTAAGGTT3′ (forward), 5′AACATCATGACAGGTCGTGAT3′ (reverse). Relative expression of *PAR-2* mRNA was calculated using 2^−ΔΔ*C*_*t*_^ method. Each test was repeated three times. According to the average expression level (2.854) of *PAR-2* in OSCC tissues, 116 patients were divided into low expression group (*n*=66) and high expression group (*n*=50).

### Cell transfection

OSCC cells in exponential growth period were used for cell transfection. PAR-2 siRNA and corresponding negative control (NC) were constructed by Genechem Co. Ltd. (Shanghai, China), and the sequences were as follows: PAR-2 siRNA: 5′-GGGCCAUCAAACUCAUUGU-3′, siRNA control: 5′-UUCUCCGAACGUGUCACGU-3′. siRNA was transfected into SCC-25 cells using Lipofectamine™2000 (Invitrogen, CA, U.S.A.) according to the manufacturer’s instruction. The cells were incubated at 37°C for 48 h, with 5% CO_2_. Then *PAR-2* mRNA level of the transfected cells was measured using qRT-PCR to investigate interfering effects. Final concentration of siRNA was 40 nmol/L, which was used for subsequent experiments.

### Cell proliferation

Cell proliferation was determined adopting MTT cell proliferation kit (Cayman Chemical) following the manufacturer’s instruction. In brief, cells transfected by PAR-2 siRNA or si-NC were seeded on 96-well plates, and cell concentration was adjusted to 2 × 10^4^ ml^−1^. They were cultured in a incubator at 37°C with 5% CO_2_ for 0, 24, 48, and 72 h, respectively. Then 50 μl MTT solution (5 mg/ml) were added into cells, and continuously incubated for 6 h. Next, of 20% SDS was added into each well, and incubation lasted overnight at room temperature. MTT enzyme-linked immunometric meter was used to measure OD value (450 nm).

### Transwell assay

OSCC cells’ migration and invasion were detected through transwell assay (Corning Glass Works, Corning, N.Y., U.S.A.) without and with matrigel (BD Biosciences), respectively. After 72 h of transfection, the cells in each group were collected and inoculated in 96-well plates, 5 × 10^4^ in each hole. 50 μl of serum-free medium with BSA was added to upper compartment. Then lower chamber received 500 μl of DMEM medium with 10% FBS. Later, 200 μl cell suspension was seeded to the upper chamber, and incubated at 37°C with 5% CO_2_ for 24 h. Cells in the bottom chamber were stained with 0.1% crystal violet for 30 min, and then counted for 10 random regions under microscope.

Meanwhile, Transwell trial coated with matrigel was used to measure the invasion of OSCC cells, according to migration analysis.

### Western blot

Transfected OSCC cells were lysed using RIPA buffer (Thermo Scientific, Belmont, MA, U.S.A.) at 4°C for 30 min. Proteins in OSCC cells were extracted and separated through 10% SDS-polyacrylamide gel electrophoresis (SDS-PAGE), and transferred onto a PVDF membrane (Roche) via electroblotting. The membranes were blocked in 5% nonfat milk for 1 h at room temperature and then incubated at 4°C overnight with primary antibodies, including anti-PI3K (ab32089), anti-p-PI3K (ab182651), anti-Akt (ab179463), anti-p-Akt (ab38449), anti-mTOR (ab2732), anti-p-mTOR (ab109268), and anti-GAPDH (ab181602) antibodies. Next, the membrane was incubated for 1.5 h at room temperature using second antibody (1:2000, Abcam, China). Target band of protein was visualized using ECL Western blotting kit (Millipore, Boston, MA, U.S.A.).

### Statistical analysis

SPSS 18.0 (SPSS Inc., Chicago, IL, U.S.A.) and GraphPad Prism (GraphPad, San Diego, CA, U.S.A.) software were used for statistical analysis and graphics, respectively. Experiments were performed at least three times and data were expressed as mean ± SD (standard deviation). Difference between two groups was compared through two-tailed Student’s *t*-test or Chi-square test. *P*<0.05 was considered statistically significant.

## Results

### Baseline characteristics of the study population

In our study, 116 patients diagnosed with OSCC were enrolled, including 64 males and 52 females. The average age of the patients was 56.57 ± 12.35 years. Of the patients, 58 had smoking history, while 56 drinking history. Metastasis was observed in 36 patients. As for TNM stage, 69 patients were grouped into stages I–II, and 47 into stages III–IV. Detailed information of the study subjects is summarized in Table 1.

**Table 1:** The correlation of *PAR-2* mRNA level with clinical characteristics of OSCC patients

Characteristics	*N* (*n*=116)	Low expression (*n*=66)	High expression (*n*=50)	*P*
Age (years)				0.485
≥60	60	36	24	
<60	56	30	26	
Gender				0.852
Male	64	33	31	
Female	52	33	29	
Smoking				0.134
Yes	58	29	29	
No	58	37	21	
Drinking				0.147
Yes	56	28	28	
No	60	38	22	
Tumor differentiation				0.037
High-middle	75	48	27	
Low	41	18	23	
Lymphatic metastasis				0.069
Yes	36	16	20	
No	80	50	30	
TNM stage				0.028
I–II	69	45	24	
III–IV	47	21	26	

### Expression level of *PAR-2* mRNA in OSCC tissues and cells

Expression level of *PAR-2* mRNA in OSCC tissues and cells was detected by RT-qPCR. The results showed that *PAR-2* mRNA level in OSCC tissue was significantly higher than that in adjacent normal tissue (*P*<0.01, Figure 1A). Similarly, compared with HOK cells, *PAR-2* mRNA expression level in OSCC cell line SCC-25 was also significantly increased (*P*<0.01, Figure 1B).

**Figure 1:** Relative expression of PAR-2 mRNA in tissues and cell lines (**A**) Expression level of *PAR-2* mRNA in OSCC and adjacent normal tissues. (**B**) Expression level of *PAR-2* mRNA in SCC-25 cells and HOK. **P<0.01.

### Association analysis of *PAR-2* mRNA level with clinical parameters of OSCC patients

According to the mean expression level of *PAR-2* in OSCC tissues, 116 OSCC patients were divided into low (*n*=66) and high (*n*=50) expression groups. Chi-square test showed that expression level of *PAR-2* mRNA was obviously correlated with low tumor differentiation (*P*=0.037) and advanced TNM stage (*P*=0.028) in OSCC, but not with age, gender, smoking drinking status, or lymphatic metastasis (*P*>0.05 for all) (Table 1).

### The influence of *PAR-2* activator PAR-2AP on OSCC cell proliferation, migration, and invasion

PAR-2AP, a special agonist for *PAR-2*, was used to treat SCC-25 cells *in vitro*, with concentrations of 0, 100, and 200 μM. The activation of *PAR-2* using PAR-2AP could significantly promote the proliferation of SCC-25 cells (**P<0.01, Figure 2A). Meanwhile, the migration and invasion of SCC-25 cells were also significantly enhanced (*P<0.05; **P<0.01; ***P<0.001, Figure 2B,C). In addition, to examine the effects of control peptide and to consolidate the specificity of PAR-2AP, SCC-25 cells were cultured for 72 h in the presence of activation peptide (PAR-2AP) or control peptide (KGLVS-NH2) at concentrations of 0, 100, and 200 μM, respectively, in serum-free culture media. Differences between PAR-2AP and control peptides groups were statistically significant at 100 and 200 μM concentrations (**P<0.01, Figure 2D). SCC-25 cells were cultured for 72 h in the presence or absence of 200 μM activation peptides or in the presence of 200 μM control peptides. The results showed that PAR-2AP could significantly enhance the migration and invasion of SCC-25 cells compared with no peptide and control peptide groups (**P<0.01; ***P<0.001, Figure 2E,F). Moreover, with PAR-2AP concentration growing, the effect of SCC-25 cells was elevated. PAR-2AP could enhance malignant behaviors of OSCC cells in a concentration-dependent manner.

**Figure 2:** The effects of *PAR-2* activation on biological behaviors of OSCC cells. SCC-25 cells were treated with PAR-2AP, an activator of *PAR-2, in vitro* with the concentrations of 0, 100, and 200 μM, respectively PAR-2AP treatment could promote the proliferation (**A**), migration (**B**), and invasion (**C**) of SCC-25 cells. Cell proliferation assays on SCC-25 cells with or without PAR-2 activation, with the former including activation peptide PAR-2AP and control peptide (**D**). The migration (**E**) and invasion (**F**) of SCC-25 cells were also more quick in PAR-2AP group than in the other two conditions. *P<0.05, **P<0.01, ***P<0.001.

### *PAR-2* knockout inhibited the proliferation, migration, and invasion of OSCC cells

To investigate functional roles of *PAR-2* in OSCC progression, interference vector specific to *PAR-2* (PAR-2 siRNA) was designed for our study. qRT-PCR showed that relative level of *PAR-2* mRNA was obviously decreased after the transfection with PAR-2 siRNA, compared with cells transfected by si-NC (*P*<0.001, Figure 3).

**Figure 3:** Relative expression of *PAR-2* mRNA was significantly down-regulated in SCC-25 cells transfected with PAR-2 siRNA ***P<0.001.

MTT result showed that the proliferation of SCC-25 cells transfected by PAR-2 siRNA was significantly decreased, compared with si-NC group (*P*<0.05, Figure 4A). Transwell trail was used to detect the influence of *PAR-2* level on the migration and invasion of SCC-25 cells. Compared with si-NC group, the number of migratory cells in PAR-2 siRNA transfection group was significantly lowered (*P*<0.01, Figure 4B). Likewise, the number of invasive cells in PAR-2 siRNA transfection group was also significantly lower than that in si-NC group (*P*<0.01, Figure 4C). The knockout of *PAR-2* could inhibit aggressive behaviors of OSCC cells *in vitro*.

**Figure 4:** Effects of PAR-2 to proliferation, migration and invasion of SCC-25 cells (**A**) *PAR-2* knockout inhibited the proliferation of SCC-25 cells. (**B**) *PAR-2* knockout could suppress the migration of SCC cells. (**C**) *PAR-2* knockout reduced the invasion of SCC cells. *P<0.05 and **P<0.01.

### *PAR-2* regulated PI3K/AKT signaling pathway in OSCC cells

In the present study, the influence of *PAR-2* level on PI3K/AKT signaling pathway in OSCC cells was explored. Western blot showed that expression levels of p-PI3K, p-AKT, and p-mTOR were significantly up-regulated in SCC-25 cells treated with 200 μM PAR-2AP (*P*<0.05, Figure 5A). On the contrary, p-PI3K, p-AKT, and p-mTOR expressions were remarkably down-regulated in SCC-25 cells transfected by PAR-2 siRNA, compared with si-NC transfection group (*P*<0.05, Figure 5B). While the expression of PI3K, AKT, and mTOR was not influenced by *PAR-2* levels, but *PAR-2* might enhance phosphorylation levels of related proteins, thus contributing to the activation of the PI3K/AKT signaling pathway in OSCC.

**Figure 5:** The effects of *PAR-2* expression on the activation of PI3K/AKT signaling pathway Excessive activation of *PAR-2* using PAR-2AP could enhance the expressions of p-PI3K, p-AKT, and p-mTOR, thus activating PI3K/AKT signaling pathway (**A**). The knockout of *PAR-2* could inhibit PI3K/AKT signaling pathway (**B**). *P<0.05.

### *PAR-2* took part in the progression of OSCC cells through PI3K/AKT signaling pathway

To explore the mechanism of *PAR-2* affecting OSCC progression, PI3K specific inhibitor LY294002 (20 μM) and AKT specific inhibitor MK2206 (20 μM) were added into OSCC cells treated with 200 μM PAR-2AP. Western blot results showed LY294002 significantly inhibited PI3K/AKT signaling pathway through suppressing the expressions of PI3K, p-PI3K, p-AKT, and p-mTOR proteins in OSCC cells treated with PAR-2AP (*P*<0.05, Figure 6). Besides, MK2206 significantly inhibited PI3K/AKT signaling pathway through suppressing the expressions of p-AKT and p-mTOR proteins in OSCC cells treated with PAR-2AP (*P*<0.05, Figure 6). Cell biological behavior analyses suggested that LY294002 could inhibit malignant proliferation, migration, and invasion of SCC-25 cells, even if the cells had excessive activation of *PAR-2* (200 μM) (*P*<0.05, Figure 7A–C). LY294002 reversed oncogenic function caused by the activation of *PAR-2* in SCC-25 cells.

**Figure 6:** LY294002 and MK2206 inhibited the activation of PI3K/AKT signaling pathway in SCC-25 cells *P<0.05.

**Figure 7:** Inhibition of PI3K/AKT signaling pathway could influence the bilogical behaviors of SCC-25 cells The addition of LY294002 could inhibit the proliferation (**A**), migration (**B**), and invasion (**C**) of OSCC cells treated with PAR-2AP. *P<0.05 and **P<0.01 indicated significant difference between the compared two.

## Discussion

OSCC is a complex malignancy affected by interactions between environmental and genetic factors. Tobacco use and alcohol consumption are two known risk factors for OSCC [20]. In addition, various susceptible genetic loci have also been identified for this disease, most seating in chromosome 9 and chromosome 17 [21]. However, those recognized factors could not explain all OSCC cases. More potentially related genetic factors need to be identified for understanding the disease transformation and progression. In the current study, we investigated the function of *PAR-2* in OSCC progression, as well as related molecular mechanisms.

*PAR-2* serves as an oncogene in various human cancers. Its over-expression might contribute to malignant progression, thus leading to poor prognosis. For instance, Wang et al. reported that the expression of *PAR-2* was obviously higher in gastric stromal tumor tissues than in adjacent normal tissues. Moreover, such elevated expression was positively correlated with tumor invasion and metastasis [22]. In esophageal squamous cell carcinoma, the up-regulation of *PAR-2* predicted advanced clinical stage and poor histological grade, possibly being a biomarker for unsatisfactory prognosis [23]. In the present study, we investigated clinical significance of *PAR-2* in OSCC. We found that the expression of *PAR-2* mRNA was significantly higher in OSCC tissues and cell lines than in non-cancerous samples. Moreover, the up-regulation of *PAR-2* was positively correlated with poor tumor differentiation and advanced TNM stage. Excessive activation of *PAR-2* predicted aggressive progression among OSCC patients. The conclusion was consistent with those from studies on other types of cancers [22,23]. However, due to the relatively small sample size, our conclusion needed to be verified in further study with extended sample size.

Cell experiments were carried out to investigate the mechanisms of *PAR-2* affecting OSCC progression. The activation of *PAR-2* using PAR-2AP could enhance the proliferation, migration, and invasion of OSCC cells. On the contrary, the knockout of *PAR-2* decreased cell proliferation, migration, and invasion. *PAR-2* could induce malignant behaviors of OSCC cells *in vitro*. The conclusion was consistent with that from the study of Al-Eryani et al. [19]. Kanemaru et al. also reported that *PAR-2* could enhance the migration of OSCC cells *in vitro* [24]. *PAR-2* might be a potential therapeutic target for OSCC.

Growing evidence has demonstrated that *PAR-2* could regulate multiple signaling pathways in tumorigenesis. In colon cancer, *PAR-2* could enhance the survival and proliferation of colon stem/progenitor cells via promoting the activation of glycogen synthase kinase-3β (GSK3β) signaling pathway [25]. Yang et al. suggested that *PAR-2* might contribute to cancer cell migration through inhibiting the expression of miR-125b, a well-known tumor suppressor miRNA [26]. Xie et al. found that *PAR-2* played an oncogenic role in pancreatic cancer by enhancing the expression of matrix metalloproteinase (MMP)-2 which is important in MAPK signaling pathway [27]. In our study, we found that *PAR-2* might activate PI3K/AKT signaling pathway, thus contributing to malignant behaviors of OSCC cells *in vitro*. The inhibition of PI3K/AKT could reverse oncogenic function induced by the over-expression of *PAR-2*. Excessive activation of PI3K/AKT signaling pathway is frequently observed in OSCC [7]. Genetic alterations leading to the activation of PI3K/AKT pathway could contribute to malignant development of OSCC. Regulatory relationship between *PAR-2* and PI3K/AKT signaling pathway has also been reported in renal cell carcinoma by Sun et al. [18]. In addition, the study carried out by Rohani et al. demonstrated that *PAR-2* regulated the production of chemokines through PI3K/AKT pathway in HOK [28]. However, Johnson et al. reported that *PAR-2* might inhibit the expression of tumor suppressor microRNAs through activating Nf-κB signaling pathway, thereby leading to OSCC progression [29]. *PAR-2* might take part in the development and progression of OSCC through multiple signaling pathways. Further related studies are still required to improve our conclusions.

In a word, the up-regulation of *PAR-2* may be positively associated with malignant characteristics of OSCC patients. *PAR-2* could enhance cell proliferation, migration and invasion through PI3K/AKT signaling pathway in OSCC.

## Abbreviations

ATCC: American type culture collection
F2RL1: coagulation factor II (thrombin) receptor-like 1
GSK3beta: glycogen synthase kinase-3beta
MMP: matrix metalloproteinase
NC: negative control
OSCC: oral squamous cell carcinoma
*PAR-2*: protease activated receptor 2
qRT-PCR: quantitative real-time PCR
